# Analysis of the Effect of Health Management of Chronic Diseases and Metabolic Disorders under the Guidance of B-Ultrasound

This article has been retracted.

**DOI:** 10.1155/2021/6648611

**Published:** 2021-02-02

**Authors:** Xiu Luo, Yi Wang

**Affiliations:** ^1^School of Health and Intelligent Engineering, Chengdu Medical College, Chengdu, Sichuan 610500, China; ^2^Department of ENT, The First Affiliated Hospital of Chengdu Medical College, Chengdu, Sichuan 610500, China

## Abstract

Chronic diseases are diseases with insidious onset, prolonged duration, and intractability and are associated with complex etiology and multiple morbidities, including hypertension, obesity, liver disease, kidney disease, cancer, cardiovascular disease, and chronic lung disease. For patients with chronic diseases, although the cause of the disease is not in the spleen and stomach, medication or further development of the disease will affect the function of the spleen and stomach disorders, leading to worsening of the disease. In this article, ultrasound is used to detect health disorders of the spleen and stomach. Patients should eat a light diet and exercise more. Elderly patients can increase abdominal massage and other health care. It should be emphasized that the prevalence of chronic diseases is not lower in people with high education or high economic income but is closely related to people's daily living habits; secondly, we should enhance physical exercise and advocate annual physical examination. Finally, we need to develop different measures according to different regions to prevent and treat chronic diseases and give timely feedback to the interventions. New preventive and curative measures are given in time to improve public health.

## 1. Introduction

Chronic diseases are diseases with insidious onset and long duration, are difficult to cure, have complex causes, and are associated with multiple morbidities, including hypertension, obesity, liver disease, kidney disease, cancer, cardiovascular and cerebrovascular disease, and chronic lung disease [1]. The World Health Organization (WHO) estimates that, in the next 10 years, approximately 388 million deaths worldwide will be due to chronic diseases, of which 80 million will be Chinese, and the economically active age group will be the majority of the population. Over the same period, at least $550 billion of China's economic losses (WHO, 2005) will be caused by three chronic diseases: stroke, heart disease, and diabetes [2]. The progress report on disease prevention and control also states that the incidence of chronic diseases in China is increasing rapidly, with cardiovascular disease, cancer, and other chronic diseases being the leading causes of death, accounting for 86.6% of all deaths in China [3], and that the mortality rate from chronic diseases in these countries is higher than that in some high-income countries. With the rapid development of society and the improvement of people's quality of life, coupled with the aging of the population, chronic diseases have become a major threat to people's health and an important risk factor for socioeconomic growth [4, 5]. For example, in China, 300 million adult males smoke and 160 million adults suffer from hypertension; in urban areas, more than 20% of minors aged 7–17 years are overweight or obese. Most chronic diseases require lifelong medication and treatment, which greatly increases the burden on society and families and impedes social development. Most chronic diseases require lifelong medication and treatment, which greatly increases the burden on society and families and impedes social development. In short, if effective measures are not taken to prevent and control chronic diseases, China's health problems will become more serious in the future [6].

Due to the social and economic development, the speeding up of the pace of life, and the increasing pressure of work, along with the emergence of high-calorie, high-fat diet and the emergence of life habits such as walking by car, the number of obese patients is increasing. At present, obesity has become a worldwide health problem. According to survey data from 1980, obese people accounted for 10% of the population, while data from 2012 show that nearly 50% of the population is currently overweight and close to obesity, with 20%–30% of obese people living in World Trade Organization countries [7–9], indicating that obesity is closely related to economic development leading to fast-paced lifestyles and changes in diet. Epidemiological studies on obesity found that, in 1996, the prevalence of obesity (BMI ≥ 28) and overweight (BMI ≥ 24) among Chinese adults was 2.48% and 18.28%, respectively, with the prevalence significantly higher in urban than in rural areas, north than south, and women than men [10]. It has been reported that the number of obese Chinese has exceeded 70 million, and the number of obese people is doubling every five years [11]. Adipositis is a risk factor for many chronic noninfectious diseases, so it is important to work actively to prevent obesity. There are three common types of obesity prevention. The first one is to eliminate risk factors leading to overweight and obesity. The second one is to avoid weight gain after weight loss. The third one is to prevent obesity from increasing after physical obesity. Weight management starts mainly with nutrition, but patient compliance is not easy. High blood pressure is one of the most common chronic diseases and the main cause for the development of cardiovascular diseases in humans. In the year 2012, 17,5 million people worldwide were affected by cardiovascular diseases, which are 31% of all deaths. These include 740 million deaths from ischemic heart disease and 6,7 million deaths from stroke, which is more than 80% of all deaths [12]. According to the Disease Surveillance System Causes of Death Surveillance data, the mortality rate of cardiovascular disease in rural areas was 229.0 per 100,000 in 2008, which was higher than that in urban areas [13]. In addition, the annual medical cost of hypertension in China is 31.89 billion RMB, of which 26.39 billion RMB is spent on outpatient care and the remaining 5.5 billion RMB is spent on hospitalization [14]. In 2002, the economic losses due to hypertension in these countries accounted for 5.61% of the total health costs in these countries [15]. One of the most effective interventions for hypertension is comprehensive community-based management. Community-based prevention and control should be based on a combination of high-risk population strategies and whole-population strategies (primary prevention with equal emphasis on secondary and tertiary prevention strategies) [16–20]. According to the Chinese Hypertension Prevention and Treatment Guidelines (2010), the prevalence of hypertension in these countries is still on the rise, with 2 out of 10 adults suffering from hypertension, but the awareness, treatment, and control rates are low. A classification of chronic diseases can be shown in Figure 1. Therefore, there is an urgent need to increase interventions for the prevention of hypertension.

Epidemiological research focuses on populations with certain characteristics, including various diseases or health states and the distribution and influencing factors of certain diseases and health states, which are all biological, physical, cultural, social, and behavioral factors affecting health. Epidemiology commonly uses the following measures to describe distribution: incidence, prevalence, prevalence, mortality, and so on. Epidemiological induction is mainly reflected in the two aspects of “description” and “analysis,” in which there is analysis in the description and analysis throughout the description [21–23]. Methods of analysis in epidemiology include observational studies, experimental studies, and mathematical modeling [24]. Among them, experimental studies are those in which a factor or measure is applied or eliminated and the effect of the factor or measure on the subject is observed. Experimental research includes three types of trials: clinical trials, field trials, and community intervention trials [25].

The paper uses ultrasound to detect splenic and gastric health disorders. In patients with chronic diseases, the cause is not in the spleen or stomach, but medicines and the progression of the disease affect the function of the spleen and stomach diseases, leading to a worsening of the disease. It should be stressed that the prevalence of chronic diseases in people with higher education or high economic incomes is not low but is closely linked to people's daily living habits. Secondly, we must strengthen the movement and commit ourselves to annual physical examinations. Finally, different regions should develop different prevention and treatment options and provide timely feedback on interventions. New preventive and therapeutic measures to improve public health are being taken in good time.

## 2. Overview of Chronic Diseases and Epidemiology

### 2.1. Liver Disease

Liver diseases are mainly due to liver disorders, including autoimmune liver disease, drug-induced liver disease, and inherited metabolic liver disease. Hepatitis B (hepatitis B virus, HBV) is the leading cause of liver disease in these countries, with the prevalence of HBV infection decreasing from 9.8% to 7.2%. It has been reported that about 2 billion people worldwide are currently infected with HBV, of which about 400 million are carriers of HBV. About 4.5 million people are newly infected each year, 25% of these people develop chronic liver disease, and about 1 million people die each year from HBV infection that leads to hepatitis or cirrhosis. Currently, there are about 110,000 people who die of liver cancer each year, and 70%–80% of these 110,000 people are infected with HBV. There are currently no multicenter, large-scale epidemiological studies related to fatty liver disease in China, and there are only a few small, targeted studies of certain special populations. The prevalence of nonalcoholic steatohepatitis in adults is estimated to be in the range of 14–31%, with 5% of patients progressing to nonalcoholic cirrhosis. The prevalence of alcoholic liver disease in these countries increased from 4.2% of liver disease in 1991 to 21.3% in 1996 and was higher in the north than in the south. As shown in Figure 2, the prevalence of alcoholic fatty liver disease, suspected alcoholic fatty liver disease, and nonalcoholic fatty liver disease was found to be 0.79%, 1.15%, and 15.35%, respectively, in the epidemiological survey of adults with fatty liver disease.

### 2.2. Chronic Respiratory Disease

Chronic respiratory diseases (COPD) are chronic diseases of the lung tissue and airways. In 2012, more than 3 million people died from COPD, accounting for 6% of global deaths, making it the fifth leading cause of death in the world, and according to the WHO, COPD is expected to rise to the fourth leading cause of death in the world by 2030. Meanwhile, a 2006–2008 survey in Hubei Province showed that respiratory diseases were the fifth leading cause of death in the population. However, due to the lack of relevant health resources, the awareness of COPD among COPD patients worldwide is still low, and the prevalence of COPD, disability, and mortality rates is underestimated, resulting in a heavy economic burden on patients, families, and society. There are two main causes of COPD: individual susceptibility factors and environmental factors, both of which influence each other. The environmental factors include occupational dust, smoking, air pollution, and bacterial infections, as shown in Figure 3. Numerous studies have shown that the occurrence of these diseases is closely related to the ambient air quality, lifestyle, and bad behavior. As for the intervention measures to prevent chronic respiratory diseases, they mainly focus on prevention, strengthening physical exercise, reducing harmful gas emissions, and building a “smoke-free” environment.

### 2.3. Chronic Cardiovascular Disease

Hypertension is a cardiovascular disease that poses a serious threat to human life and health, with complex and diverse pathogenesis, high morbidity, disability, and mortality rates, costing the country a large amount of medical and social resources and bringing a heavy economic burden to people and their families. Hypertension is one of the most common chronic diseases and an important factor in the development of cardiovascular disease. In 2012, cardiovascular diseases accounted for 17.5 million deaths worldwide or 31% of all deaths, including 740 million deaths from ischemic heart disease and 6.7 million deaths from stroke, accounting for more than 80% of all deaths. According to data from the China Disease Surveillance System for Causes of Death, the mortality rate from cardiovascular diseases in rural areas was 229.0 per 100,000 in 2008, which was higher than that in urban areas. In addition, the annual medical cost of hypertension in China is 31.89 billion RMB, of which 26.39 billion RMB is spent on outpatient care and the remaining 5.5 billion RMB is spent on hospitalization. In 2002, the economic losses due to hypertension in these countries accounted for 5.61% of the total health costs. One of the most effective interventions for hypertension is comprehensive community-based management. Community-based prevention and treatment should be based on a combination of high-risk population strategies and population-wide strategies (primary prevention and secondary and tertiary prevention strategies). According to the Chinese Hypertension Prevention and Treatment Guidelines (2010), the prevalence of hypertension in these countries is still on the rise, with 2 in 10 adults suffering from hypertension, but the awareness, treatment, and control rates of hypertension are low. Therefore, there is an urgent need to increase interventions to prevent hypertension.

Diabetes mellitus is a systemic metabolic disorder characterized by persistent hyperglycemia due to multiple causes of metabolic disorders, characterized by inadequate secretion and/or dysfunction of insulin, mainly impaired glucose metabolism and associated sugars, and protein and fat metabolism leading to multiple organs and ultimately impaired dysfunction. Diabetes mellitus includes type I diabetes, type II diabetes, pregnancy diabetes, and other types of diabetes. Type I diabetes is caused by the destruction of the autoimmune system and insufficient insulin secretion and often begins in childhood or adolescence, so type I diabetes requires insulin injection. Type II diabetes is a metabolic disease that is 85% to 95% of the diabetic population, mainly caused by insulin deficiency and resistance to insulin.

After cardiovascular and cerebrovascular diseases and cancer, diabetes has become the third largest chronic noncommunicable disease threatening human health. In the 1990s, according to the International Diabetes Federation (IDF), there were approximately 100 million diabetics in the world; by 2007, this number had rapidly increased to 246 million, and it is expected that by 2025, 380 million people worldwide will suffer from diabetes. In these countries, the number of diabetics will continue to increase as the population ages. Because most people with diabetes have a long disease course, gradually as the disease progresses, they may experience damage to certain organs throughout the body, and eventually, in severe cases, they may become disabled or even die as a result of complications of diabetes. According to the Diabetes Prevention and Treatment Guidelines, the prevalence of diabetes is higher in urban than in rural areas and higher in economically developed areas than in less developed areas, which may be related to the lifestyle and eating habits of people in developed areas, economic status, and other factors. In addition, according to different regions, the prevalence of diabetes has ethnic characteristics, and the prevalence of diabetes differs among different ethnic groups in the same region; for example, the prevalence of diabetes in Hui in Ningxia Autonomous Region is higher than that in Han, and the prevalence of diabetes in Han in Inner Mongolia Autonomous Region is higher than that in Mongolian. In short, diabetes has become a major public health problem of global concern, which brings not only pain to patients but also a heavy burden to families and society. Therefore, it is crucial to understand the causes of diabetes prevalence in a timely manner and to develop effective prevention and treatment measures.

## 3. Ultrasound-Guided Metabolic Management of Chronic Diseases

In this part, the application of cardiac ultrasound in the diagnosis of hypertensive heart disease helps improve the detection rate of cardiac abnormalities, improve the accuracy of diagnosis results, and promote the development of relevant therapeutic work. When blood pressure rises, the function of the heart will be greatly affected, and the heart is an important organ that causes blood pressure to fall or rise; if patients are not diagnosed and treated in time, it may lead to heart failure, ventricular dilation, other symptoms, and even death.

### 3.1. Diagnosis of Cardiovascular Disease

Hypertension is a common clinical disease that is difficult to cure. When patients are under hypertension for a long period of time, it is easy to cause symptoms such as abnormal heart function and myocardial hypertrophy, thus leading to hypertensive heart disease, which is not conducive to a good life and may even threaten patients' health. The production of hypertension is closely related to the patient's psychology, sleep, living habits, diet, and other factors. In recent years, the incidence of hypertension is increasing year by year and developing in a younger direction, due to the aging process and changes in people's lifestyles and dietary habits in these countries. Therefore, this condition should be diagnosed and treated as early as possible in order to reduce the risk of the disease, avoid further deterioration, and ensure the safety of the patient's life. In the past, electrocardiogram (ECG) was often used to diagnose this condition. As a noninvasive examination method, ECG has less impact on the patient's function; therefore, this examination method is more frequently used in clinical practice. In the past, ECG was often used as a noninvasive examination method, which had less influence on patient's function, and therefore, this examination method was used more frequently in clinical practice, thus effectively ensuring patient safety.

In addition, ultrasound is popular with patients because it is repeatable and very inexpensive. During the examination, ultrasound has a better understanding of the anatomical structure of the heart and can fix the image development, which facilitates the smooth development of subsequent observation, as shown in Figure 4. For patients with hypertensive heart disease, long-term exposure to high blood pressure will result in different degrees of damage to heart function, and cardiac ultrasound can emit ultrasound waves through the probe to the location of the heart without causing any damage to the heart. Cardiac activity is helpful in the formulation of the next treatment plan. If the patient has ventricular hypertrophy, but the ECG still shows normal results due to potential offset, it is easy to miss or misdiagnose, which is not conducive to the effective development of treatment. Therefore, when diagnosing hypertensive heart disease clinically, cardiac ultrasound examination can be used to improve the accuracy of diagnosis and provide a scientific basis for the formulation of treatment plans, so as to avoid further development of the patient's condition and reduce the danger and mortality of the disease.

In the present study, the detection rate of cardiac abnormalities in the research group was 96.67%, which was higher than that of the control group (73.33%), and the difference was statistically significant (*P* < 0.05). In this regard, ultrasound examination can be applied in the clinical diagnosis of hypertensive heart disease to ensure the correctness of clinical diagnosis and reduce the occurrence of misdiagnosis and omission, so as to ensure the scientific and rational nature of the treatment plan. The accuracy of diagnostic results in the research group was 66.67%, which was significantly lower than that in the control group (93.33%), and the difference was statistically significant (*P* < 0.05); thus, it can be seen that the accuracy of ultrasound in diagnosing patients' heart rhythm or heart rate changes, left ventricular strain hypertrophy, myocardial ischemia, and left atrial enlargement is higher, which to a certain extent can provide greater convenience for the related treatment work. Compared with ECG examination, cardiac ultrasound has greater sensitivity and specificity. It can effectively check the blood flow condition of the heart through the scanner, provide a scientific basis for heart function judgment, and help improve the accuracy of diagnosis. In summary, the application of cardiac ultrasound in the diagnosis of hypertensive heart disease can effectively improve the detection rate of cardiac abnormalities, improve the accuracy of diagnosis results, and promote the development of relevant therapeutic work.

### 32. Liver B-Ultrasound Imaging Evaluation

Forty-four patients were selected who were hospitalized for liver disease at our hospital from April 2018 to December 2019. Inclusion criteria included the following: meeting the clinical diagnostic criteria for chronic liver disease in these countries; fatty liver disease diagnosed by liver ultrasound; BPRS score less than 40; age 18 to 65 years. Exclusion criteria included the following: comorbid viral hepatitis and other types of liver diseases; chronic alcohol users; other concomitant serious physical diseases. The patients were randomly divided into an exercise group of 22 patients and a control group of 22 patients using a data map. The two groups of patients were compared in terms of general information (see Figure 5), and there was no statistically significant difference (*P* > 0.05). Both groups were treated with antipsychotic drugs and routine psychiatric care.

For fatty liver, both groups were treated symptomatically with liver-protective drugs and dietary control. Exercise therapy was also added to the observation group as follows: (1) Exercise plan was formulated. Aerobic exercise started from low intensity and low volume and then the volume and intensity of exercise gradually increased; the heart rate after exercise was about 60% of the maximum heart rate. The patient's compliance to exercise is increased by the use of appropriate words and small gifts. The purpose and function of exercise were explained to patients, and appropriate use of words and small gifts was made to increase patients' compliance to exercise. The patients were placed in supine, left lateral, and right lateral lying positions, and the morphology, borders, size, structure, and spot intensity of the liver were recorded to diagnose fatty liver and classify the disease condition. In this paper, SPSS22.0 was used to process the data. Measurement data were described by (*x*− ± *s*), and *t*-test was used for comparison between groups; count data were described by frequency, and *X*^2^ test was used for comparison between groups. The rank-sum test was used for rank data. The test level *α* = 0.05.

Fatty liver disease is a pathological condition resulting from excessive accumulation of liver fat. According to surveys, the prevalence of fatty liver disease is significantly higher in schizophrenia patients with prolonged hospitalization than in normal subjects, which is closely related to the use of antipsychotic medications and reduced daily activity levels. Fatty liver can promote liver damage in schizophrenic patients and therefore should be actively intervened. In this study, we used exercise therapy for long-term hospitalized schizophrenia patients and liver B-ultrasound imaging to evaluate the effect of the intervention on patients with fatty liver disease. As shown in Figure 5, the results showed that the degree of fatty liver in the exercise group was significantly reduced and the BMI value was significantly lower than that in the control group after the intervention. This suggests that exercise therapy can effectively improve the effect of intervention on fatty liver in hospitalized schizophrenia patients and effectively reduce BMI and has a positive significance in reducing liver damage.

### 3.3. Chronic Disease Information Management

Individuals with chronic disease generally experience a lower quality of services, which negatively impacts all aspects of life, such as poor employment and worsening health outcomes. Chronic disease places a heavy economic burden on society, reducing the quality of life for more than one billion people, who may be at risk for reduced functional capacity and disability. Chronic diseases have become the pandemic of our time, accounting for more than 50% of health care expenditures, and are the leading cause of death. Existing models of chronic disease management are poorly structured, as evidenced by poor adherence by patients with chronic diseases and poorly controlled outcomes of treatment. Mobile health technologies can engage patients and provide more models of chronic disease management such as treatment options, care, management, and multiple hybrid models. By providing effective, coordinated, and personalized models that reduce costs and improve the quality of care, mHealth provides tremendous support for controlling the epidemic of chronic disease. A number of systematic evaluation/meta-analysis studies have found that mHealth technologies can improve functional capacity in patients with chronic diseases. It is important to summarize the results to understand under which circumstances and what types of mHealth technologies are effective in decision-making for patients and clinicians. This study analyzed a systematic evaluation/meta-analysis of mHealth technologies for the management of chronic diseases to evaluate the effectiveness of mHealth technologies compared to standard care or no intervention for the management of chronic diseases and to evaluate the impact of mHealth technologies on the physical and functional abilities of patients with chronic diseases.

The AMSTAR and PRISMA scales are used to evaluate the methodological and reporting quality of the evidence. Based on the evaluation results, the effectiveness of mHealth technology on different diseases and populations with different characteristics of the same disease was analyzed and summarized to provide the best therapeutic support measures for medical workers and patients and to reduce the burden on medical workers and families caring for patients, as shown in Figure 6. A total of 500 questionnaires were distributed, and 481 questionnaires were returned, with a return rate of 96.2%.

There were 247 female subjects in this survey, accounting for 51.4% of the total number of subjects, with a relatively reasonable composition of men and women; the largest number of subjects, 67.6% of the total, was between 21 and 45 years old; their educational level was concentrated in college/undergraduate level, accounting for 44.3%. The main mode of payment for medical expenses is urban residents' medical insurance. The majority of survey respondents were employees of enterprises and public institutions, accounting for 53.2% of the total number of survey respondents. 66.7% of the survey respondents believed that their health condition was relatively good based on their usual performance. 51.7% of the 481 survey respondents believed that they were relatively knowledgeable about mHealth technology. 88.4% of the survey respondents believed that mHealth technology was convenient and fast, and 317.4% of the survey respondents believed that it was convenient and fast. Of the 316 survey respondents, 77.3% said that mHealth technology could provide online consultation services, 72.3% said that mHealth technology could provide information about fitness and exercise, and 66.3% said that mHealth technology could provide health care services. Mobile applications were the most frequently used mobile health technology category, followed by wearable devices.

When it comes to health issues, 72.6% of respondents would prefer to visit a doctor and 50.9% would prefer to consult a health website or medical app. 275 respondents would prefer to use mobile health technology for information about diseases, medications, and recent medical advice. Of the respondents' intention to use mHealth, 389 indicated that they intended to start or continue using mHealth. 379 respondents predicted that they would use mHealth in the next few months. 76.1% of respondents indicated that they would like to continue using mHealth in the future. 76.7% of respondents indicated that they would recommend mHealth to others and 73.2% of the respondents indicated that they would recommend mHealth to others. In addition, 64.2% of the study participants said they would recommend mHealth technology to the elderly, 64.2% would recommend it to patients with chronic diseases, and more than half would recommend it to parents of infants and toddlers.

## 4. Results and Discussion

This study shows that the awareness rate of mHealth management technology among patients with chronic diseases is 51.7% (249/481), but about 80% of them indicated that they would continue to use mHealth technology or plan to start using it, indicating that the use of mHealth products is not high among the general public and most people do not have the concept of using mHealth technology to manage their health, as shown in Figure 7. With the rapid development of science and technology, a series of new technologies such as artificial intelligence are increasingly applied in the public's life, and the public will tend to choose to rely on online medical services for initial consultation and basic medical care information. Chronic diseases include cardiovascular and cerebrovascular diseases, cancer, chronic respiratory diseases, diabetes, and kidney disease.

Chronic diseases, such as the common cold, are a serious threat to the health of the population and have developed into a major health care problem affecting the country's economic and social development. The occurrence and prevalence of chronic diseases are closely related to demographic, behavioral, environmental, economic, and social factors. As industrialization and urbanization in these countries accelerate, the aging of the population affects people's lifestyles, ecological environment, and food safety situation and gradually has a profound impact on the incidence of chronic diseases, the prevalence of chronic diseases, and the increase in the number of deaths caused by chronic diseases, and the burden of chronic diseases becomes increasingly heavy. In 2016, the WHO reported that communicable diseases and chronic noncommunicable diseases continue to plague many countries, especially in developing countries, and called on countries around the world to take more favorable health care measures to comprehensively address the threats posed by these two types of diseases.

The report called on countries around the world to adopt more favorable health care measures to comprehensively address the threat of these two major types of diseases. The number of people under management was 88.35 million, the number of people with diabetes was 26.14 million, and the premature mortality rate for major chronic diseases was 19.1% in 2013. In the Report on Nutrition and Chronic Diseases (2015), it is stated that chronic disease monitoring includes disease monitoring (chronic disease and nutrition monitoring, cause of death monitoring, and cancer follow-up registration); environmental health hazard monitoring (urban and rural drinking water sanitation, rural environmental sanitation, public places health hazards, air pollution and other health effects on the population, and human biology monitoring); key population health monitoring (student health risk factors and monitoring of common diseases). At the same time, we are actively promoting the transfer of scientific and technological achievements and the promotion and application of appropriate technologies, including the transfer of health scientific and technological achievements and the promotion of appropriate technologies in primary health care services.

Chronic diseases have complex etiology, long duration, many complications, and heavy treatment burden, but residents' awareness of chronic diseases and self-care management is low. Patients with chronic diseases need to reduce complications and improve health outcomes through long-term self-management, good treatment adherence, and positive changes in poor lifestyle habits.

Nonalcoholic fatty liver disease (NAFLD) is a disease characterized by the presence of 5% fat in the liver and affects more than 1 billion people worldwide. With the globalization of Western lifestyles and the obesity epidemic, the incidence of metabolic syndrome and T2DM has increased, as has the prevalence of NAFLD, which has become the leading cause of chronic liver disease. It has become a very common disease in developed countries and has been increasing in the past decades.

The prevalence of obesity is associated with an increase in obesity, and obese people are now making 50% to 80% of obese patients. In the past, obesity alone was considered good and reversible. However, the presence of other etiologies can link the progression of fattyosis. Fattyosis exacerbates liver damage, so it promotes oxidation, causes inflammation, increases susceptibility to apoptosis, promotes the progression of fibrosis, and eventually leads to cirrhosis and even liver failure and liver cancer. NAFLD is a liver symptom of metabolic syndrome. NAFLD is therefore associated not only with an increase in liver mortality but also with an increase in overall mortality, especially in cardiovascular and malignant tumors. It is therefore necessary to precisely quantify its range and monitor its dynamics. Until now, the characteristic clinical symptoms, signs, and test criteria for NAFLD have not been identified, so it is very important to find a simple means of early diagnosis. NAFLD has certain pathological features in relation to hepatic biopsy, but it is usually diagnosed as a diagnosis of exclusion, and hepatic biopsies have known limitations such as variability and invasiveness of the samples.

Due to the relatively high prevalence of NAFLD/NASH in the general population, liver biopsies are not suitable for mass screening. Computed tomography is known to detect hepatic steatosis at moderate to severe levels as a means of reducing liver attenuation. The sensitivity and specificity of liver/spleen CT ratio (L/S) for the diagnosis of fatty liver can reach 82% and 100%, respectively, and its diagnostic accuracy is better than that of ultrasound, as shown in Figure 8. However, CT uses ionizing radiation and is therefore not suitable for widespread use in asymptomatic patients. Magnetic resonance imaging-based studies have fat content accuracy but are expensive and difficult to deploy in the large population of NAFLD. Conventional ultrasound (BUS) is the most commonly used technique to assess hepatic steatosis due to its accessibility and low cost. In addition, ultrasound can be easily performed in conscious patients, which is an advantage when imaging pediatric patients or adults who cannot tolerate MRI without sedation.

However, plain ultrasound is less accurate and subject to intra- and interobserver variability in fatty degeneration and is usually not feasible in patients with a high body mass index. Although many articles have investigated the diagnostic efficacy of conventional imaging modalities and ultrasound methods for NAFLD, there is a lack of literature on quantitative ultrasound methods for hepatic steatosis. With advances in technology, a new reference index has been defined using ultrasound attenuation principles based on instantaneous elastography (Fibro Scan): the Controlled Attenuation Parameter (CAP), which is highly correlated with steatosis and allows for a qualitative diagnosis of steatosis. The purpose of this study was to compare three methods of fatty liver diagnosis, explore the superiority of Fibro Scan in fatty liver diagnosis, and provide a new test for screening, early diagnosis, treatment, and follow-up of fatty liver.

## 5. Conclusion

In this paper, ultrasound was used to detect splenic and gastric health disorders. In patients with chronic diseases, the cause is not in the spleen or stomach, but medicines and the progression of the disease affect the function of the spleen and stomach diseases, leading to a worsening of the disease. It should be stressed that the prevalence of chronic diseases in people with higher education or high economic incomes is not low but is closely linked to people's daily living habits. Secondly, we must strengthen the movement and commit ourselves to annual physical examinations. Finally, different regions should develop different prevention and treatment options and provide timely feedback on interventions. New preventive and therapeutic measures to improve public health are being taken in good time.

## Figures and Tables

**Figure 1:** Chronic disease classification.

**Figure 2:** Epidemiological investigation of fatty liver in adults.

**Figure 3:** Respiratory chronicity.

**Figure 4:** Effectiveness of ultrasound in the diagnosis of cardiovascular disease.

**Figure 5:** Fatty liver intervention effect.

**Figure 6:** Ultrasound-based therapeutic adjuncts for chronic diseases.

**Figure 7:** Health management techniques for chronic diseases.

**Figure 8:** Comparison of the effects of ultrasound-guided chronic disease management.

## Data Availability

The data used to support the findings of this study are available from the corresponding author upon request.
